The article "Ghrelin Regulates Cyclooxygenase-2 Expression and Promotes Gastric Cancer Cell Progression" was published in 2021. Journal: Comput Math Methods Med.

# Ghrelin Regulates Cyclooxygenase-2 Expression and Promotes Gastric Cancer Cell Progression

**DOI:** 10.1155/2021/5576808

**Published:** 2021-05-22

**Authors:** Huanqing Li, Xiaohong Zhang, Li Feng

**Affiliations:** Endoscopy Center, Minhang District Central Hospital of Fudan University, Shanghai, China

## Abstract

**Aim:**

To research the molecular mechanism of ghrelin in apoptosis, migratory, and invasion of gastric cancer (GC) cells.

**Methods:**

After GC AGS cells were handled with ghrelin (10^–8^ M), cyclooxygenase-2 inhibitor NS398 (100 *μ*M), and Akt inhibitor perifosine (10uM), the rates of apoptosis were detected by TUNEL assay and flow cytometry assay. We assessed the expressions of PI3K, p-Akt, and COX-2 proteins by making use of Western blot analysis. The cell migratory and invasion were detected by using wound-healing and transwell analysis.

**Results:**

The migratory and invasion were increased in ghrelin-treated cells, while the rates of apoptosis were decreased. GC AGS cells treated with ghrelin showed an increase in protein expression of p-Akt, PI3K, and COX-2. After cells were treated with Akt inhibitor perifosine, the protein expression of p-Akt, PI3K, and COX-2 and the cell migratory, invasion, and apoptosis were partly recovered. After cells were treated with cyclooxygenase-2 inhibitor NS398, the protein expression of COX-2 and the cell migratory and invasion were decreased, while the rates of apoptosis were increased.

**Conclusion:**

Ghrelin regulates cell migration, invasion, and apoptosis in GC cells through targeting PI3K/Akt/COX-2. Ghrelin increases the expression of COX-2 in GC cells by targeting PI3K/Akt. Ghrelin is suggested to be one of the molecular targets in GC.

## 1. Introduction

Cancer is a leading cause of people's death worldwide. Among all these cancers, gastric cancer (GC) is one of the leading widespread oncological diseases. Although the detection rate and the cure rate of early GC are increasing, the 5-year survival rate of developing GC is still very low [1]. The mechanism of developing GC involves many signaling pathways, the cyclooxygenase-2 (COX-2) and prostaglandin E2 (PGE-2) pathway included [2].

The conversion of arachidonic acid to several prostaglandins is catalyzed by cyclooxygenase (COX). The main isoforms of cyclooxygenases are COX-1 and COX-2. COX-1 has been found for expression in most tissues, involving gastric mucosal blood flow and renal blood flow. COX-2 has been known as an inducible enzyme, which is highly expressed after the body is stimulated by inflammatory factors. The pathological mechanism of GC induced by H. pylori includes morphological changes caused by the interaction of bacteria and host, such as atrophic gastritis and gastrointestinal metaplasia mediated by COX-2 overexpression [3]. Studies show that through making use of the COX-2 inhibitor, treatment of trefoil factor 1-deficient mice reduces the size of the gastric adenomas [4]. It has been indicated from recent studies that the COX-2 inhibitor has a preventive influence on Helicobacter pylori-associated GC [5, 6].

As we all know, ghrelin is a peptide produced in the stomach, which can regulate gastric acid secretion and gastric motion [7–11]. Ghrelin could be extracted from the gastric mucosa and acted through its receptors: GHSR. Besides, the evidence is showing the effect of ghrelin in apoptosis, migration, and invasion [12]. But the exact molecular mechanism of ghrelin in GC is still unclear.

Our recent studies have shown that ghrelin can reduce apoptosis by targeting MAPKs/iNOS and Akt/eNOS in hepatocytes [13], and ghrelin regulates autophagy by targeting PI3K/Akt/Bcl-2 in mice [14]. In this research, we examined the molecular mechanism of ghrelin in the development of GC cells.

## 2. Materials and Methods

### 2.1. Materials

Ghrelin was bought from ProSpec (Ness Ziona, Israel). Perifosine, an Akt inhibitor, was bought from Keryx Biopharmaceuticals (New York, NY, USA). We bought NS398, a cyclooxygenase-2 inhibitor, from Cayman Chemical Company (Ann Arbor, MI, USA). We bought antibodies against PI3K, p-Akt, COX-2, and actin from Santa Cruz Biotechnology Inc. (Dallas, TX, USA).

### 2.2. Cell Culture and Treatment

The AGS cells were bought from the American Type Culture Collection (Rockville, MD, USA). We cultured the cells in RPMI-1640 culture medium (Thermo Fisher Scientific, Waltham, MA, USA). We passaged cells every 5 days by washing twice. AGS cells were treated with ghrelin dissolving into 10^−8^ *μ*M/L, Akt inhibitor perifosine dissolving into 10 *μ*M/L, and the cyclooxygenase-2 inhibitor NS398 dissolving into 100 *μ*M/L through RPMI-1640 medium.

We divided cells into four groups: normal control group, ghrelin group, perifosine group (ghrelin+Akt inhibitor perifosine), and NS398 group (ghrelin+cyclooxygenase-2 inhibitor NS398+Akt inhibitor perifosine). Perifosine was added into cells 24 hours after being treated with ghrelin in the AGS cells. NS398 was added into cells 24 hours after being treated with perifosine in the AGS cells.

### 2.3. Western Blot Analysis

RIPA buffer and protease inhibitor lysed the AGS cells. The concentrations of protein were tested through the BCA method. Protein was uncoupled with SDS-PAGE. We transferred it to PVDF. Then, we incubated the material with antibodies, including PI3K (1 : 1000), COX-2 (1 : 1000), p-Akt (1 : 1000), and actin (1 : 1000). The proteins were tested by the Western blot analysis [15].

### 2.4. Flow Cytometry

We collected AGS cells after they were handled with NS398, perifosine, and ghrelin and washed twice. The cells were mixed with propidium iodide and annexin V-fluorescein isothiocyanate and waited for 15 min. Then, the rates of apoptosis were analyzed through flow cytometry [16].

### 2.5. TUNEL Assay

After AGS cells were treated with NS398, perifosine, and ghrelin, the cells were collected and washed twice. The cells were treated with proteinase K, TUNEL, and DAPI dyes. Then, cells were mixed for 1 hour. The rates of apoptosis were analyzed through TUNEL assay (Kaiji Biotech, Nanjing, China) [17].

### 2.6. Transwell Assay

Transwell assay was used for analyzing the invasion of AGS cells. 1 × 10^5^ AGS cells got ready in medium without serum. The upper chamber prepared with Matrigel was plated with 100 *μ*L of AGS cell suspension. Then, the lower chamber was plated with 20% serum. The invasion cells were analyzed by three random fields at a magnification of 200.

### 2.7. Wound-Healing Assay

We made use of a wound-healing assay aiming at analyzing migratory AGS cells. A pipette tip was used to scratch the confluent cells in a six-well plate. PBS was used to wash the plate, and a new medium was added. After 24 hours, the cell migration was analyzed.

### 2.8. Analysis of Statistics

We made use of SPSS 20.0 statistical analysis software (IBM-SPSS, Inc., Chicago, IL, USA) for statistical comparison. We analyzed differences among groups with analysis of variance, and Bonferroni's *t*-test followed. All experiments were repeated at least three times, and the data were expressed as the mean standard deviation (SD). The significance of statistics was considered with *P* < 0.05.

## 3. Results

### 3.1. Ghrelin Regulated the Apoptosis, Invasion, and Migration in GC Cells

Aiming at studying the molecular mechanism of ghrelin in GC cells, we cultured AGS cells in the RPMI-1640 culture medium, and they were treated with ghrelin dissolving into 10^−8^ *μ*M/L. To test the apoptosis induced by ghrelin, we used TUNEL assay and flow cytometry. In the flow cytometry assay, apoptotic cells' percentage in the control group and the ghrelin group was 7.81% ± 0.97% and 5.16% ± 0.24% (^∗^*P* < 0.05) (Figures 1(a) and 1(b)). In the TUNEL assay, apoptotic cells' percentage in the control group and the ghrelin group was 0.88% ± 0.12% and 0.37% ± 0.14% (^∗^*P* < 0.05) (Figures 2(a) and 2(b)).

To test the migratory induced by ghrelin in GC cells, we used a wound-healing assay. Results showed that ghrelin significantly increased migratory compare to the control group (^∗^*P* < 0.05) (Figures 3(a) and 3(b)).

To test the invasion induced by ghrelin in GC cells, we used a transwell assay. Results showed that ghrelin significantly increased invasion in comparison with the control group, averaging 208 cells versus 159 cells per six random microscopic fields (^∗^*P* < 0.05) (Figures 4(a) and 4(b)). All these results above demonstrated that ghrelin could reduce apoptosis and increase migration and invasion in GC cells.

### 3.2. Ghrelin Regulated the Expression of Cyclooxygenase-2 by Targeting PI3K/Akt in GC Cells

After AGS cells were treated with ghrelin (10^–8^ M) and perifosine (Akt inhibitor, 10 *μ*M), we analyzed the protein expressions of p-Akt, PI3k, and COX-2 through Western blot analysis. GC AGS cells treated with ghrelin showed an increase in protein expression of p-Akt, PI3K, and COX-2. After cells were treated with perifosine (Akt inhibitor), the protein expression was recovered (*P* < 0.05) (Figure 5). All these results above demonstrated that ghrelin regulated the expression of cyclooxygenase-2 by targeting PI3K/Akt in GC cells.

### 3.3. Ghrelin Regulated the Apoptosis, Invasion, and Migration in GC Cells by Targeting PI3K/Akt and COX-2

Our results had demonstrated that ghrelin could reduce apoptosis and increase invasion and migration in GC cells. The results of flow cytometry analysis showed that with the ghrelin group as the control, the apoptosis rate of the perifosine group increased (Figure 1(c)). Taking the perifosine group as a control, the apoptosis of the NS398 group increased (Figure 1(d)). The results of the TUNEL assay showed that with the ghrelin group as the control, the apoptosis of the perifosine group increased (Figure 2(c)). Taking the perifosine group as a control, the apoptosis of the NS398 group increased (Figure 2(d)), which was consistent with the results of flow cytometry analysis. Wound-healing test analysis results showed that compared with the ghrelin group, the cell migration of the perifosine group was significantly increased (Figure 3(c)). Compared with the perifosine group, the cell migration of the NS398 group was significantly increased (Figure 3(d)). Compared with the ghrelin group, the cell invasion ability of the perifosine group was significantly reduced (Figure 4(c)); compared with the perifosine group, the cell invasion ability of the NS398 group was significantly reduced (Figure 4(d)). In summary, GC AGS cells treated with ghrelin showed that protein expression of PI3K, p-Akt, and COX-2 increased. After cells were treated with Akt inhibitor perifosine, the protein expressions of p-Akt, PI3K, and COX-2 and the migration, invasion, and apoptosis were partly recovered. After cells were treated with cyclooxygenase-2 inhibitor NS398, the protein expression of COX-2 and the cell migration and invasion were decreased, while the rates of apoptosis were increased. All results above demonstrated that ghrelin regulated the apoptosis, invasion, and migration in GC cells by targeting PI3K/Akt/COX-2.

## 4. Discussion

GC is one of the high-mortality diseases and it is the fifth most common cancer and the third most common cause of cancer death in the world [18]. There are many mechanisms in the occurrence and development of GC. But the exact molecular mechanism is still unclear [19]. It is currently considered that surgery is the only radical treatment for GC. With the advancement of surgical techniques and the implementation of traditional radiotherapy, chemotherapy, and neoadjuvant therapy, progress has been made. The main treatment for advanced gastric cancer is a combination of neoadjuvant radiotherapy and chemotherapy, molecular targeted therapy, and immunotherapy [20]. Therefore, more effective drugs are urgently needed for GC. However, the role of ghrelin and its relationship to COX-2 in GC have not been investigated, though ghrelin is secreted mainly from the stomach.

Our previous research confirmed that miR-21 mediated ghrelin's inhibitory effect on ethanol-induced apoptosis of gastric epithelial cells [21]. Ghrelin has been found to regulate apoptosis, invasion, and metastasis in glioma cells and gastric cancer cells, including the AMPK and GHS-R/NF-*κ*B pathway [22, 23]. Otherwise, ghrelin can induce colon adenocarcinoma cells' apoptosis by proteasome inhibition and autophagy [24]. Our research showed that cell migration and invasion were increased in ghrelin-treated cells, while the rates of apoptosis were decreased. These researches show that ghrelin regulates GC cell progression.

Phosphoinositide 3-kinase (PI3K) signal pathway is one of the most common changes in human cancer, which has a paramount function in the occurrence and development of a tumor. Some researches have shown that ghrelin increases proliferation and metastasis in cancer cells through targeting PI3K/AKT/mTOR [25–27]. However, the mechanism of the antiapoptotic effects of ghrelin is not clear and requires further investigation. The mechanism of ghrelin in anticancer effects induced by NS398 has not been reported in GC. Our researches showed that GC AGS cells treated with ghrelin showed that protein expression of COX-2 goes up. After cells were treated with perifosine, the protein expression of COX-2 was partly recovered. These results suggest that ghrelin regulates the expression of cyclooxygenase-2 by targeting PI3K/Akt in GC cells.

As a specific COX-2 inhibitor, NS398 has a chemopreventive influence on gastrointestinal cancer [28, 29]. Gastrin acts on cyclooxygenase-2 expression of human GC cells induced by cholecystokinin receptor through the JAK2/STAT3/PI3K/Akt pathway [30]. A selective COX-2 inhibitor has an antitumor effect on GC cells, which may be partly mediated by the downregulation of Akt in the mitochondrial apoptosis pathway [31]. The high expression of COX-2 is beneficial to the occurrence and metastasis of GC [32]. Our researches showed that GC AGS cells treated with ghrelin showed that protein expression of COX-2 went up. Otherwise, our results had demonstrated that ghrelin could reduce apoptosis and increase migratory and invasion in GC cells. The protein expression of COX-2 and the migration, invasion, and apoptosis were partly recovered after cells were handled with cyclooxygenase-2 inhibitor NS398. All these results above demonstrate that ghrelin regulates the apoptosis, migration, and invasion in GC cells by targeting PI3K/Akt/COX-2.

This study has a limitation. This study only investigated the role of ghrelin in one GC cell line. In future research, we will explore the mechanism of ghrelin in more GC cell lines. In addition, we also plan to further study in animal models.

Our study has made an investigation on the underlying mechanisms of ghrelin and its relationship to COX-2, though it is not the first one to prove these effects induced by ghrelin. Ghrelin is suggested to be one of the molecular targets in GC.

## 5. Conclusion

The migration, invasion, and apoptosis in GC cells are regulated by ghrelin through targeting PI3K/Akt/COX-2. The expression of COX-2 in GC cells is regulated by ghrelin through targeting PI3K/Akt. Ghrelin is suggested to be one of the molecular targets in GC. To our knowledge, this is the first report on the biological mechanism by which ghrelin regulates the development of gastric cancer by targeting PI3K/Akt/COX-2. The results of this study provide a theoretical basis for ghrelin as a potential therapeutic drug for GC.

## Figures and Tables

**Figure 1:** The rates of apoptosis were analyzed through flow cytometry. ^∗^*P* < 0.05: the ghrelin group in comparison with the control group; ^&^*P* < 0.05: the perifosine group in comparison with the ghrelin group; ^#^*P* < 0.05: the NS398 group in comparison with the perifosine group.

**Figure 2:** The rates of apoptosis were analyzed through TUNEL assay (Kaiji Biotech, Nanjing, China). Apoptotic cells' percentage depended on TUNEL assay. The magnification was ×200. ^∗^*P* < 0.05: the ghrelin group in comparison with the control group; ^&^*P* < 0.05: the perifosine group in comparison with the ghrelin group; ^#^*P* < 0.05: the NS398 group in comparison with the perifosine group.

**Figure 3:** Wound-healing assay was used for analyzing migratory of AGS cells. The magnification was ×100. ^∗^*P* < 0.05: the ghrelin group in comparison with the control group; ^&^*P* < 0.05: the perifosine group in comparison with the ghrelin group; ^#^*P* < 0.05: the NS398 group in comparison with the perifosine group.

**Figure 4:** Transwell assay was used for analyzing invasion of AGS cells. The magnification was ×200. ^∗^*P* < 0.05: the ghrelin group in comparison with the control group; ^&^*P* < 0.05: the perifosine group in comparison with the ghrelin group; ^#^*P* < 0.05: the NS398 group in comparison with the perifosine group.

**Figure 5:** The proteins were tested with the Western blot analysis. ^∗^*P* < 0.05: the ghrelin group in comparison with the control group; ^&^*P* < 0.05: the perifosine group in comparison with the ghrelin group; ^#^*P* < 0.05: the NS398 group in comparison with the perifosine group.

## Data Availability

The datasets used and/or analyzed during the current study are available from the corresponding author on reasonable request.
